The article "Association between Single Nucleotide Polymorphism rs9891119 of STAT3 Gene and the Genetic Susceptibility to Type 2 Diabetes in Chinese Han Population from Guangdong" was published in 2021. Journal: J Healthc Eng.

# Association between Single Nucleotide Polymorphism rs9891119 of STAT3 Gene and the Genetic Susceptibility to Type 2 Diabetes in Chinese Han Population from Guangdong

**DOI:** 10.1155/2021/6657324

**Published:** 2021-03-24

**Authors:** Haibing Yu, Xuyun Xu, Jialu Huang, Jian Xu, Hao Liu, Yuxun Xie, Chunwen Lin, Congcong Pan, Danli Kong, Yuanlin Ding

**Affiliations:** ^1^Department of Epidemiology and Health Statistics, School of Public Health, Guangdong Medical University, Dongguan, Guangdong Province 523808, China; ^2^Shantou Hospital of Traditional Chinese Medicine, Shantou, Guangdong Province 515031, China

## Abstract

**Background:**

The aim of this study was to investigate the association between single nucleotide polymorphism (SNP) rs9891119 of the signal transducer and activator of the transcription 3 (STAT3) gene and genetic susceptibility to type 2 diabetes in Chinese Han population from the Guangdong province.

**Objective:**

The aim of the present study was to explore the relationship between single nucleotide polymorphism rs9891119 of STAT3 gene and type 2 diabetes mellitus (T2DM), which provides a basis for molecular genetic research on the pathogenesis of T2DM in Chinese Han population.

**Methods:**

In our case-control study, the SNP rs9891119 was picked out from the STAT3 gene and the SNP genotyping was performed by using the SNPscan^™^ kit in 1092 patients with type 2 diabetes as cases and 1092 normal persons as controls. The distributions of genotype and allele frequencies in two groups were analyzed by SPSS 20.0 software.

**Results:**

Our results showed that the alleles of A and C of rs9891119 of the STAT3 gene were 54.3 and 45.7% in patients with type 2 diabetes, while 55.5% and 44.5% in the normal persons, which have no statistical significance (*P* > 0.05). There were also no significant differences in AA, AC, and CC genotype frequencies between type 2 diabetes patients and normal persons. There were no significant differences in codominant, dominant, recessive, and overdominant genetic models of SNP rs9891119 before and after adjusting the covariant factors (*P* > 0.05).

**Conclusions:**

Therefore, genetic susceptibility to type 2 diabetes may be not associated with SNP rs9891119 of the STAT3 gene in Chinese Han population from the Guangdong province.

## 1. Introduction

As one of the most common endocrine and metabolic diseases, diabetes is severely harmful to human health. Type 2 diabetes patients make up 95% of cases of diabetes. In 2020, approximately 463 million people worldwide suffer from diabetes, and, in 2019, 4.2 million people died of the disease and its complications [1]. Studies have reported that type 2 diabetes is a kind of complex chronic disease, caused by the interaction of genetic and environmental factors, often appearing in familial hereditary tendency, and more than one-third of type 2 diabetes patients have family diabetes history [2].

The article "Association between Single Nucleotide Polymorphism rs9891119 of STAT3 Gene and the Genetic Susceptibility to Type 2 Diabetes in Chinese Han Population from Guangdong" was published in 2021. Journal: J Healthc Eng.

Leptin is a hormone produced primarily in the adipocytes of the white adipose tissue [3] and is the key biomarker of the adipose tissue [4], which is closely related to obesity, diabetes, and metabolic syndrome [5–8]. The study found that elevated serum leptin levels contribute to the development of metabolic complications of obesity, especially diabetes and insulin resistance [9–12]. JAK/STAT is considered to be the main pathway for leptin signaling in pathways that regulate appetite and energy metabolism [13]. STAT3 plays an important role in the JAK/STAT signal-mediated leptin pathway [13, 14]. Previous studies reported that there are many genes associated with type 2 diabetes in the leptin signaling pathways including STAT3, playing a regulator role in the signal transduction of various cytokines, growth factors, and hormones, which are involved in the regulation of body growth and immune responses. Moreover, STAT3 is recognized as a key regulator of insulin resistance [14] and conducts the regulation of appetite and energy metabolism by monitoring the transcription of downstream target genes [15–18]. Previous studies have found that STAT3 in the nerve center of knockout mice can lead to obesity, diabetes, and energy imbalance [19].

Based on previous studies of the research group, the SNP RS9891119 of the STAT3 gene was selected in this study. The SNPscanTM kit is used to investigate SNP rs9891119 of the STAT3 gene in the leptin signaling pathway between type 2 diabetes patients and normal persons in Chinese Han population from Guangdong. This study aims to evaluate whether these polymorphisms are associated with type 2 diabetes and provide a valuable reference for molecular genetics research of type 2 diabetes in Chinese Han population from Guangdong.

## 2. Subjects and Methods

### 2.1. Research Subjects

In our case-control study, 1092 patients with confirmed type 2 diabetes were selected in 10 hospitals from Shenzhen, Donguan, Maoming, Zhanjiang, and Shaoguan of the Guangdong province. Type 2 diabetes was diagnosed under the criteria of the World Health Organization (WHO) in 1999. The inclusive criteria of type 2 diabetes patients are as follows. (1) Range of age 20–70 years; (2) random blood glucose levels ≥11.1 mmol/L with diabetes symptoms including polydipsia, polyphagia, polyuria, weight loss, itchiness, blurred vision, and other acute metabolic disorders caused by hyperglycemia and fasting blood glucose levels ≥7.0 mmol/L without diabetes symptoms; blood glucose levels ≥11.1 mmol/L with a glucose tolerance test two hours after the oral dose; (3) without malignancies, cardiovascular diseases, kidney diseases, and other severe interference diseases. Moreover, 1092 normal persons were also selected as the control group after body checks in the same 10 hospitals. The inclusive criteria of normal persons are as follows: (1) rang of age 20–70 years; (2) without family history of diabetes; (3) healthy after physical examination including medical history, blood glucose, and other biochemical test results [20]. The study was approved by the Ethics Committee, and all the participants were fully informed about the procedures and risks involved in the research. All surveys and samples have obtained the consents of participants in advance, and the informed consent forms had legally consented. All the participants were the permanent residents of Han nationality in the Guangdong province, and there is no kinship among them.

The article "Association between Single Nucleotide Polymorphism rs9891119 of STAT3 Gene and the Genetic Susceptibility to Type 2 Diabetes in Chinese Han Population from Guangdong" was published in 2021. Journal: J Healthc Eng.

### 2.2. Field Investigation

Standardized questionnaires were designed to collect the clinical trial information by the investigators. According to the inclusion criteria, we would collect the basic information of subjects including age, gender, and native place and their clinical data including disease history, course of disease, smoking history, family history, and complications. After the investigation, height, weight, and right-arm blood pressure were measured by trained personnel in duplicate, and the results were averaged. The body mass index (BMI) was calculated as weight (kg) divided by the square of height (m^2^). About 5 ml peripheral blood samples were collected in early morning for detecting clinical biochemical indications. Fasting plasma glucose (FPG) was detected by the hexokinase method. Total cholesterol (TC), triglyceride (TG), high-density lipoprotein cholesterol (HDL-C), and low-density lipoprotein cholesterol (LDL-C) were measured by enzymatic methods. Glycosylated hemoglobin A1c (HbA1C) was determined by high-performance liquid chromatography. Other biochemical parameters were detected by the automatic biochemical analyzer.

### 2.3. DNA Preparation

Peripheral venous blood (2 mL) collected from each subject was put into an anticoagulant tube with ethylenediaminetetraacetic acid disodium salt-Na_2_ (k2-EDTA). The DNA was extracted by the salting-out method after digestion with Proteinase K and stored in a −80°C refrigerator.

### 2.4. SNP Selection and Genotyping

The tag SNP (MAF > 0.05 and *r*^2^ ≥ 0.8) was selected from the STAT3 gene and its range of 5 kb using with the HapMap website, a public database (http://www.hapmap.org) and Hapoloview (version 4.2). The potential function of tag SNP was predicted using FastSNP (http://fastsnp.ibms.sinica.edu.tw/pages/input_CandidateGeneSearch.jsp), and SNP rs9891119 located in the intron1 of the STAT3 gene was identified with high predicted score. Based on previous research experience, this paper selected the rs3754219 site of the GLUT1 gene. SNP rs9891119 of the STAT3 gene was genotyped using the SNPscan^™^ kit ^18^. Specific experimental steps are as follows. (1) Detection of DNA quality and concentration: run a DNA sample (1 *μ*l) on the 1% agarose gel. (2) Sample lysis: take 4 *μ*L of DNA samples into 96-well plates, mix with 2.5 *μ*L 4 × DNA lysis buffer and 3.5 *μ*L distilled water, centrifuge after covering with parafilm, incubate in the PCR machine at 98°C for 5 min, and then store in the ice immediately. (3) Adapter ligation reaction: add 10 *μ*L premix solution to DNA lysis samples, shaking slightly after covering with film, centrifuge for 30 s at 3000 rpm, and transfer to the PCR machine with four cycles at 94°C for 1 min and 58°C for 4 h, then 2 min hold at 4°C, and at 72°C forever. (4) Multiplex polymerase chain reaction: take 1 *μ*L of the ligation product into a new 96-well plate and mix with 19 *μ*L PCR premix solution, centrifuge for 30 s at 3000 rpm after covering and shaking, and transfer to the PCR machine to carry out. (5) DNA sequencing: take 1 *μ*L of the PCR product after diluting 10 times, mix with 0.5 *μ*L Liz500 SIZE STANDARD and 8.5 *μ*L Hi-Di, and carry out denaturation at 95°C for 5 min. The DNA sequencing was performed using an ABI3130XL sequencer. (6) Data analysis: the experimental data were analyzed using GeneMapper 4.1 (Applied Biosystems, USA) to obtain the fluorescent labeling and length of the PCR product and the corresponding gene information of the SNP site and allele.

The article "Association between Single Nucleotide Polymorphism rs9891119 of STAT3 Gene and the Genetic Susceptibility to Type 2 Diabetes in Chinese Han Population from Guangdong" was published in 2021. Journal: J Healthc Eng.

### 2.5. Statistical Analysis

Software SPSS 20.0 was used to analyze the experimental data. The chi-square test and *t*-test were applied to compare the general information, genotype, and allele frequency of the two groups. The conditional logistic regression analysis was applied to calculate the OR and 95% CI after adjusting the factors including age and BMI. The chi-square goodness-of-fit test was used to test the distribution of the genotype in Hardy–Weinberg equilibrium. Measurement data was expressed by mean ± standard deviation (*x* ± *s*). *P* < 0.05 was considered as the level of statistical significance.

## 3. Results

### 3.1. General Situation

A total of 1092 patients with type 2 diabetes and 1092 normal persons were enrolled in this study. Excluding individuals with the SNP missing rate higher than 20%, 1067 cases and 1054 controls were finally included for subsequent statistical analysis. In the case group, there were 532 males and 535 females, aged 59.71 ± 11.87 years, while in the control group, there were 532 males and 522 females, aged 57.23 ± 10.41 years. There were significant differences in the age composition, body mass index, fasting blood glucose, triglyceride levels, and low-density cholesterol between the two groups. The age composition, body mass index, fasting blood glucose, and triglyceride levels of the case group were higher than the control group. However, low-density lipoprotein cholesterol of the case group was lower than that of the control group, as shown in Table 1.

### 3.2. Comparison between SNP rs9891119 Genotype and Allele Frequency

The distribution of alleles in the case group and control group is shown in Table 2. The A and C allele frequencies in SNP rs9891119 were not significantly different between the two groups (*P* > 0.05). There were also no significant differences in AA, AC, and CC genotype frequencies between the two groups (*P* > 0.05), which suggested that SNP rs9891119 of the STAT3 gene might be not associated with genetic susceptibility to type 2 diabetes.

### 3.3. Comparison of Two Genetic Models

There are no significant differences in codominant, dominant, recessive, and overdominant genetic models of SNP rs9891119 before and after adjusting the covariant factors including age and body mass index, as shown in Table 3.

## 4. Discussion

Caused by complex interactions of multiple factors, including the interaction of genetic and environmental factors [21, 22], type 2 diabetes is a chronic disease characterized by decreased secretion of insulin by the pancreas and resistance to the action of insulin in various tissues, hyperglycemia, and relative complications due to absolute or relative insulin deficiency or insulin resistance [23]. Type 2 diabetes is severely harmful to the health of mankind, which could cause damage, dysfunction, and failure to tissues and organs including eyes, kidneys, cardiovascular, and nervous systems. Therefore, more and more research studies are devoted to finding out the important internal factors leading to their pathogenesis. Genetic factors, especially its susceptibility genes and polymorphisms, are gradually demonstrated in the in-depth study.

Leptin can affect many metabolic pathways of the human body and plays an important role in maintaining the normal metabolic balance. It may lead to a series of symptoms associated with type 2 diabetes via various pathways, which includes insulin resistance and hyperinsulinemia. The level of plasma leptin is influenced by many factors including gender, age, body fat distribution, free fatty acids, glucocorticoids, and insulin. The level of insulin plays a crucial role in leptin regulation and negative feedback regulation that exists between leptin and insulin. Leptin is considered as the intermediary of the “fat and insulin axis,” which is involved in the regulation of insulin secretion. Decrease of leptin can reduce the sensitivity of insulin, and insulin can stimulate leptin secretion. Therefore, leptin and insulin affect each other in the production mechanism, and their interaction participates in the genesis and development of many diseases such as type 2 diabetes [24]. The molecular basis of the leptin signaling pathway is attributed to the molecular structure, functional status level, and expression levels of STAT3 and Janus kinase 2 (JAK2) proteins in leptin targeting cells. Decrease of expression levels of STAT3 and JAK2 proteins or their abnormal changes in the molecular structure and functional status can lead to the block of leptin signaling and inhibit the basal insulin secretion [25]. Several studies have confirmed that STAT3 is a key regulatory factor of insulin resistance and has a close contact with the occurrence and development of type 2 diabetes [26, 27]. However, the studies of STAT3 gene polymorphism, insulin resistance, and type 2 diabetes are comparatively insufficient. Tomas and others reported that SNP rs9891119 of the STAT3 gene was not associated with insulin resistance, but it provides no further explanation whether it was irrelevant with type 2 diabetes [28]. However, Jamshidi and other studies found that SNP rs2293152 of the STAT3 gene was associated with insulin resistance, but it has not confirmed its association with the occurrence and development of type 2 diabetes [29].

The article "Association between Single Nucleotide Polymorphism rs9891119 of STAT3 Gene and the Genetic Susceptibility to Type 2 Diabetes in Chinese Han Population from Guangdong" was published in 2021. Journal: J Healthc Eng.

In this study, we analyzed the SNP rs9891119 of the STAT3 gene and genetic susceptibility to type 2 diabetes involved in the leptin signaling pathway in Chinese Han population from Guangdong and explored whether there is a correlation between them. To the best of our knowledge, this is the first report about the relationship between SNP rs9891119 of STAT3 gene and type 2 diabetes. We have investigated the SNP rs9891119 of 1092 patients with type 2 diabetes and 1092 normal persons in Chinese Han population from Guangdong. The genotype analysis results of rs9891119 of the STAT3 gene showed that the frequencies of A and C alleles of rs9891119 were 54.3% and 45.7% in the patients with type 2 diabetes, while 55.5% and 44.5% in the normal persons, respectively. The genotype frequency and allele frequency were not significantly different between before and after adjusting (*P* > 0.05), suggesting that SNP rs9891119 of the STAT3 gene might not be directly related to type 2 diabetes in Chinese Han population from Guangdong.

## 5. Conclusion

This study suggests that the polymorphism of rs9891119 of the STAT3 gene is not related to the susceptibility to type 2 diabetes in Chinese Han population from Guangdong. However, it is limited for the research samples only from Han nationality in the Guangdong province, so it could not temporarily define that SNP rs9891119 of the STAT3 gene is not associated with genetic susceptibility to type 2 diabetes.

## Figures and Tables

**Table 1:** Comparison of baseline data between cases and controls.

Parameters	T2DM (*n* = 1067)	Control (*n* = 1054)	*t*/*χ*^2^	*P*
Male (%)	532(49.86)	532(50.47)	0.08	0.080
Age (years)	59.71 ± 11.87	57.23 ± 10.41	5.12	<0.001
BMI (kg/m^2^)	24.60 ± 3.24	23.58 ± 3.33	7.15	<0.001
FPG (mmol/L)	10.46 ± 4.50	5.60 ± 1.60	33.22	<0.001
TC (mmol/L)	5.31 ± 1.59	5.43 ± 1.27	-1.92	0.056
Triglyceride (mmol/L)	2.24 ± 1.03	1.31 ± 0.96	21.51	<0.001
HDL-C (mmol/L)	1.35 ± 0.54	1.37 ± 0.42	-0.95	0.398
LDL-C (mmol/L)	2.73 ± 1.04	3.03 ± 0.65	-7.98	<0.001
Hypertension (%)	396(37.11)	380(36.05)	0.26	0.257
Heart rate (bpm)	76.40 ± 15.26	76.20 ± 10.92	0.35	0.682

Note: BMI (Body Mass Index) is a person's weight in kilograms divided by the square of height in meters.

**Table 2:** Comparison of the distribution of genotype and allele frequency between the cases and controls (*n* (%)).

Group	*n*	Genotype			Allele	
		AA	AC	CC	A	C
Case	1067	315 (29.5)	529 (49.6)	223 (20.9)	1159 (54.3)	975 (45.7)
Control	1054	323 (30.6)	524 (49.7)	207 (19.7)	1170 (55.5)	938 (44.5)

**Table 3:** Comparison of genetic models between the controls and cases.

Group	Codominant			Dominant		Recessive		Overdominant	
	A/A	A/C	C/C	A/A	A/C + C/C	A/A + A/C	C/C	A/A + C/C	A/C
Control	323	524	207	323	731	847	207	530	524
Case	315	529	223	315	752	844	223	538	529
OR (95% CI)	1	1.04 (0.85–1.26)	1.10 (0.86–1.41)	1	1.05 (0.88–1.27)	1	1.08 (0.87–1.34)	1	0.99 (0.84–1.18)
*P*		0.73	0.573		0.572		0.473		0.95
adOR (95% CI)	1	1.07 (0.87–1.31)	1.10 (0.85–1.41)	1	1.08 (0.99–1.30)	1	1.05 (0.85–1.31)	1	1.03 (0.86–1.22)
ad*P*		0.734	0.58		0.45		0.644		0.752

ad: after adjusting for covariates including age and BMI.

## Data Availability

The data used to support the findings of this study are available from the corresponding author upon request.
